This article has been retracted.

# Analysis of College Students' Mental Health Education Model Based on Media Integration

**DOI:** 10.1155/2022/7381483

**Published:** 2022-09-09

**Authors:** Yanjun Wu, Shuai Jiang, Liling Zhang

**Affiliations:** ^1^School of Urban Construction, Hebei Normal University of Science and Technology, Qinhuangdao 066000, China; ^2^School of Physical Education and Health, Hebei Normal University of Science and Technology, Qinhuangdao 066000, China; ^3^School of Food Technology, Hebei Normal University of Science and Technology, Qinhuangdao 066000, China

## Abstract

At present, the mental health problems of college students in China are on the rise. Many incentives lead to college students becoming a psychological vulnerable group, lacking the minimum “decompression ability” in the face of pressure. With the emergence of new media and the increasingly obvious fusion of new media and traditional media, the recognition algorithm of media fusion begins to enter people's vision, and multimedia fusion has gradually formed an irresistible development trend. Based on the media fusion recognition algorithm under the background of media fusion, this paper studies the model of college students' mental health education. In the process of comparing the accuracy of college students' mental health, the accuracy of this method is the highest, up to 99.25%, followed by the decision tree algorithm, up to 80.53%, and finally the ant colony algorithm, up to 75.25%. Therefore, this method is more conducive to the study of college students' mental health. Under the media fusion recognition algorithm, colleges and universities should give full play to the advantages of media fusion, broaden the path of mental health education, enhance the effectiveness of mental health education, improve the quality and efficiency of education, and guide the mental health growth of college students.

## 1. Introduction

In recent years, the proportion of college students dropping out or dropping out due to various mental health problems has increased year by year. Suicide often occurs due to various emotional problems, academic stress, or interpersonal barriers. Everyone has different views on things at different ages. Especially the 16-28 year-old teenagers, once they break the bottom line, the pressure from various aspects will lead to extreme behavior. Everyone has different ways to deal with and cope with stress, but they can be divided into two types: positive and negative [1]. In the process of everyone's life, no matter how the world develops and changes, they should face it positively and optimistically and learn to communicate with others to reduce their own pressure. Because people are social animals, without communication, they will become autistic and self-closed [2, 3]. At present, most college students were born after the national reform and opening up and grew up in the period of rapid economic development. Their material conditions are gradually improving, and their brothers and sisters are also decreasing. It can be said that most students have hardly experienced any setbacks. When they encounter setbacks in their study, life, and feelings, students will be at a loss. At present, the mental health problems of college students in China are on the rise. High academic demands, low family socioeconomic status, and low self-esteem are all significant predictors of anxiety and stress in students. Drink use is a significant risk factor for college students, particularly for females. Many incentives lead to college students becoming vulnerable groups of mental health. They lack the minimum “ability to reduce pressure” in the face of pressure, resulting in a lack of motivation in the face of pressure and a tragedy that should not happen. People from all walks of life must pay full attention to this issue from the perspective of cognition and action, help the “favored son of heaven” to stay away from “depression” and regain a sunny and healthy mentality. They will lose confidence in life and feel the meaning of life. Most students can only accept praise and approval, but cannot accept the pertinent criticism and help from the people around them. However, in the face of the severe employment situation and the opportunities and challenges brought about by the reform of employment distribution system, students have not been prepared for setbacks. As the reserve force of the national talent reserve, college students are more likely to have psychological problems or obstacles due to academic pressure, employment pressure, family expectation and self-expectation, the contradiction between ideal and reality, the conflict between Chinese and Western cultures, and other pressures and influences. The old and new systems change. Numerous emotional issues, academic strain, or interpersonal hurdles frequently lead to suicide. At different ages, everyone has varying perspectives on many issues. Once they breach the bottom line, particularly among 16 to 28-year-old youths, pressure from many sources will result in severe behavior [4, 5]. Stabilizing healthy behaviors, feelings, and thoughts requires maintaining good mental health and managing any mental health issues. Focusing on mental health care can boost productivity, improve our self-perception, and strengthen bonds with others. Finally, what cannot be ignored is that we should mobilize a wider range of social forces; use television, radio, newspapers, magazines, and other media to widely publicize mental health knowledge; and set up special columns, hotlines, and consulting services to improve college students' mental health awareness. With these powerful guarantees, our mental health education can be truly implemented. The psychological status of only child college students is as follows: emotional vulnerability, poor psychological endurance, weak social ability, loneliness, strong attachment, excessive self-esteem, poor cooperation ability, easy to produce anxiety, etc. Some only children even engage in simple labor related to their own lives. A college student's success and ability to succeed academically might be affected by mental health issues. A lack of motivation and difficulties concentrating are caused by poor mental health and might result in unsatisfactory grades. The secret to students' academic achievement may lie in the availability of campus-wide services for mental illness for them to access.

With the emergence of new media and the increasingly obvious integration of new media and traditional media, media fusion recognition algorithm has also begun to enter people's vision, and multimedia fusion has gradually formed an irresistible development trend [6]. With the help of newspaper, radio, television, and Internet technologies, media fusion recognition algorithms are becoming more and more similar. Educators should consciously and systematically cultivate students' media literacy and enhance their ability to resist bad information. College students with mental health have strong ability of emotion management and regulation. They are emotionally stable, optimistic, energetic, and full of hope for life and the future. Be able to correctly express and control emotions, reasonably vent emotions, and correctly deal with joy, anger, sadness, joy, and other emotions in life [7, 8]. “New field based on media fusion recognition algorithm” “The possibility of existence has been obtained, which has also led to profound changes in communication channels. If the emergence of online media has irresistibly changed people's original lifestyle and aesthetic concepts, and naturally formed new aesthetic principles, the development and popularization of mobile media will also create a new aesthetic platform for people, build new aesthetic values, and change people's aesthetic world [9, 10].

College students' mental health is an important group in the media integration environment. At the same time, they also have a very complex psychological basis. Various religious forces try to infiltrate colleges and universities with the help of network media, which poses a serious threat to the ideological security field of colleges and universities [11]. Students' difficulties are not only economic difficulties, but also their mental health problems, which deserve high attention. Economic conditions affect and limit its growth. Low self-esteem and excessive self-reproach make some students unable to get out of the shadow of family economic situation. The fierce conflicts among rural students make them more vulnerable to disappointment and frustration, resulting in tension, anxiety, and sensitivity. The media fusion recognition algorithm has been recognized by all college students. It has become an important way for them to obtain information and the main tool for interpersonal communication. It has a certain impact on the way of thinking and mental health of college students [12]. They lack the minimum “ability to reduce pressure” in the face of pressure, resulting in a lack of motivation in the face of pressure and a tragedy that should not happen. All sectors of the society must pay full attention to this problem from the perspective of cognition and action, help the “favorite of heaven” to stay away from “depression” and regain a sunny and healthy mentality [13]. In the process of school psychological education consultation, it is undoubtedly very important to identify students' various psychological problems timely and accurately, and then take correct and targeted educational consultation measures. Under the media fusion recognition algorithm, colleges and universities should give full play to the advantages of media fusion, broaden the path of psychological education, enhance the effectiveness of psychological health education, improve the quality and efficiency of education, and guide the healthy growth of college students [14].

The innovations of this paper are as follows

1. This paper compares the characteristics of various media fusion recognition algorithms. Media fusion recognition algorithm is a new pattern under the diversified development of information transmission. It effectively combines traditional media such as newspapers and TV stations with new media communication channels such as handheld intelligent terminals and computer terminals, centralizes processing, shares resources, derives various forms of information products, and then spreads them to the audience by relying on various platforms
2. This paper analyzes and discusses the mental health standards of college students. The self-management and control of college students' emotions is not only an important part of their physical and mental health, but also a necessary condition for their self-development and personality growth. It is also the basis for them to face setbacks and adapt to the environment. Whether a person's emotions are stable and optimistic is the main symbol of a person's mental health. Students have the ability to monitor and reinforce their own behavior or skill improvement through the practise of self-management. Additionally, they are able to actively participate in their own education, get fast feedback, and develop their independence thanks to this

The overall structure of this paper consists of five parts.

The first chapter introduces the background and significance of college students' psychological education, and then introduces the main work of this paper. The second chapter mainly introduces the related work of college students' psychological education. The third chapter introduces the media fusion recognition algorithm and college students' mental health standards. The fourth chapter analyzes the mental health status of college students, carries out experiments, and draws conclusions. The fifth chapter is a summary of the full text.

## 2. Related Literature

In recent years, scholars have made special research on college students' psychological education and put forward corresponding theories. Both methodological research and empirical research have achieved fruitful research results and enriched the theoretical and practical experience of college students' mental health education. The details are as follows.

The self-management and control of college students' emotions is not only an important part of their physical and mental health, but also a necessary condition for their self-development and personality growth. It is also the basis for them to face setbacks and adapt to the environment. The network infrastructure of colleges and universities is becoming more and more perfect, which provides favorable conditions for college students to use the network. Most college students cannot resist the complicated information. Huang proposed that “mental health is a state without disease” [15]. This concept of mental health, which is only put forward from the perspective of biomedicine, has dominated people's understanding of health for a long time. The Concise Encyclopedia Britannica also defines health as “a state without disease, malnutrition, and weakness”. People once believed that as long as there was no physical disease and pain, they were healthy, and completely ignored the cultivation of healthy psychological quality [16]. Xu conducted a questionnaire survey, case interview, and other research on college students' frustration, and proposed and answered how college students should deal with frustration and how to adjust themselves after frustration from both theoretical and empirical aspects [17]. Mei defines mental health as follows: “The so-called mental health refers to the development of a person's mental state to the best within the range of incompatibility between physical, intellectual, and emotional health and the mental health of others. Ding pointed out that the school environment has an important impact on college students. For freshmen, they are faced with unfamiliar campuses and unfamiliar and closely related groups of freshmen [18]. Most students leave home for the first time, leaving their long-term dependent parents and familiar environment, which means that they will start to live independently from today and have to solve many problems by themselves [19]. Lee and Mi-na in the process of mental health education, teachers should first master various communication technologies, constantly improve media literacy, use various new media to keep close contact with students, understand the psychological characteristics of college students, reveal the laws of their psychological changes, and truly become their guide [20]. Han et al. put forward that “human nature is not an inherent abstraction of a person. In reality, it is the sum of all social relations”. Human needs include survival needs, enjoyment needs, activities, and development needs. This theory emphasizes the essence of human sociality. No one can exist independently of society [21]. Kankan et al. proposed that although most students can try to rebuild their self-rejected by reality and reestablish their life goals, some students try to avoid conflicts with reality, or vent their dissatisfaction with reality through attacks, or become extremely decadent, do not seek progress, indulge in fun and indulgence, and some students even have the idea of suicide. Xueyan put forward the main tasks of current college students' mental health education, defined the main contents, and made clear provisions on the principles, ways, and methods of college students' mental health education, as well as team building and organization management. It can be seen that the cultivation of college students' mental health and psychological quality has become one of the goals of quality education in colleges and universities [22]. It is an important part of higher education. This is a major measure for the transition from examination oriented education to quality education and the training of cross century talents [23]. Goldman et al. put forward that mental health refers to a continuous mental state. In this case, the parties can make good adaptation, have vitality, and give full play to their physical and mental potential. In various studies, health includes physical health and mental health [24].

Based on the media fusion recognition algorithm, this paper studies the mode of college students' mental health education. Educators should consciously and systematically cultivate students' media literacy and enhance their ability to resist bad information. College students with mental health have strong ability of emotion management and regulation. They are emotionally stable, optimistic, energetic, and full of hope for life and the future. Be able to correctly express and control emotions, reasonably vent emotions, and correctly handle emotions such as joy, anger, sadness, and joy in life. The early youth has the characteristics of childhood in some aspects, while the late youth has the characteristics of adulthood in some aspects. This kind of transformation often makes young people in the contradictions between childishness and maturity, dependence and independence, emotion and rationality, blindness and consciousness, ideal and reality. If these conflicts and contradictions are not effectively guided and reasonably resolved, they will form psychological conflicts and obstacles over time. Under the media fusion recognition algorithm, new requirements are put forward for all media workers. They should not only spread information and news, but also guide college students to make fair and just value judgments on various events, truthfully and objectively reflect social conditions and public opinion, and complete their glorious mission. Seeing problems is often one-sided and subjective, coupled with psychological vulnerability. Once they encounter temporary setbacks and failures, they tend to be discouraged and timid. In front of teachers, they often hide their true emotions and do not want to easily reflect their true psychological state. Impulsivity and internalization interweave together, making college students have a strong psychological conflict at this stage. At the same time, various religious forces are hovering on the edge of the law, trying to infiltrate universities with the help of Internet media, and even compete for future talent resources, so as to achieve the purpose of dividing and Westernizing China. The development of media integration has opened up a new way for mental health education in colleges and universities, and will also face many new situations and problems. Although the contents, forms, and means of education are increasingly diversified, some measures and strategies in traditional psychological education have irreplaceable advantages. The media fusion recognition algorithm poses a serious threat to the ideological foundation, self-confidence, and cohesion of college students, the formation of socialist core values and the ideological security construction of colleges and universities. Therefore, it is necessary to strengthen the religious reverse osmosis work in the media integration environment and build a long-term mechanism to prevent the infiltration of religious forces.

## 3. Methods

### 3.1. Media Fusion Recognition Algorithm

Media convergence is the trend of functional integration in the development of various media. Under the media fusion recognition algorithm, on the premise that improving the cultural soft power has gradually become an important strategic background in China, on the one hand, we can see the determination of college students' mental health education model, on the other hand, we can also see the gap between college students' mental health education model and other developed countries. Through networks, information exchange, and communication, soft power is developed. Culture has always been a powerful force, but where it once served as a guiding light for hard power, it now serves as a foundation for soft power, making it even more crucial to comprehend. The concept of media fusion recognition algorithm can be understood from both broad and narrow perspectives; in a broad sense, media fusion recognition algorithm is the combination, aggregation, and fusion of all media and their related elements [25]. Among them, integration is not only reflected in the formal level, but also in the media functions, means of communication, organizational structure, and many other aspects. In a narrow sense, media fusion refers to the fusion and qualitative change of different media forms, and finally forms a new media form. The media fusion recognition algorithm includes the combination, fusion, and even fusion of all media and their related elements, including not only the fusion of media forms, but also the fusion of communication means, media functions, organizational structure, ownership, and other elements [26]. The whole algorithm process is divided into three parts, including data acquisition and preprocessing, feature extraction, model training and recognition. The flow of the psychological health problems identifies based on media fusion consists of different process. First, the student accesses the internet in the online sequences to analyze the basic psychological characteristics. The statistical method is trained by differed psychological behavior to identify the psychological score. Then the psychological data consists of performance data and consumption data in the network log as shown in Figure 1.

The main idea of media fusion recognition algorithm is: firstly, randomly select *K* sample points from the sample set and take them as the center of the cluster. Then, according to the distance between each sample and the *K* centroids, it is divided into the nearest clusters, and then the centroids of each cluster are recalculated. Recall that *c* squared is equal to the sum of a squared and *b* squared. So, finding the square root of a squared plus *b* squared is required in order to calculate the distance *c* between a certain location and a centroid. The mean of each cluster's data points is then used to compute centroids for each cluster. After obtaining the new centroids, calculate the distance between each data point and all the centroids, and then assign the data point to the cluster with the closest centroid. The calculation formula is shown as follows:

(1) $$\begin{array}{c} d\left(x,C_{i}\right)=\sqrt{\overset{m}{\underset{j=1}{\sum }}\left(x_{j}-C_{ij}\right)}. \end{array}$$

Where

*x* is the data object,

*C*_*i*_ is the *i* cluster center,

*m* is the dimension of the data object,

*x*_*j*_ and *C*_*ij*_ are the *j* attribute values of *x* and *C*_*i*_.

The error square calculation formula of the whole data set is shown as follows:

(2) $$\begin{array}{c} SSE=\overset{k}{\underset{i=1}{\sum }}\underset{x\in C_{i}}{\sum }\left|d\left(x,C_{i}\right)\right|. \end{array}$$

Select the best attribute to split by calculating the information gain, and the attribute with the largest information gain after division is the best attribute. Information theory includes the idea of information entropy. It indicates how much information is available about an event. In general, an event will include less information the more certain or deterministic it is. Information is, to put it another way, an increase in entropy or uncertainty. Entropy is measured between 0 and 1, and Gini impurity is measured between 0 and 0.5. Consequently, we may say that Gini Impurity is superior to entropy for choosing the finest features. The information gain is calculated on the basis of information entropy, and the information entropy is calculated as shown in following:

(3) $$\begin{array}{c} \text{Entropy}\left(D\right)=-\overset{m}{\underset{i=1}{\sum }}p_{i}\log. \end{array}$$

Where

*m* represents the number of categories in the data set *D*, and.

*p*_*i*_ represents the probability of *i* category. The smaller the value, the higher the purity of *D*.

Add weight |*D*^*υ*^|/|*D*| to each branch node. When the data set is divided by attribute *a*, the information gain of sample set *D* can be calculated according to the formula.

(4) $$\begin{array}{c} \text{Gain}\left(D,a\right)=\text{Entropy}\left(D\right)-\overset{V}{\underset{\upsilon =1}{\sum }}. \end{array}$$

Firstly, the information gain of attributes is calculated, and the attributes whose information gain is higher than the average are selected, and then the attributes with the highest gain rate are selected for division.

(5) $$\begin{array}{c} \text{Gain}\_\text{ratio}\left(D,a\right)=\frac{\text{Gain}\left(D,a\right)}{\text{SI}\left(a\right)}. \end{array}$$

Among

(6) $$\begin{array}{c} \text{SI}\left(a\right)=-\overset{V}{\underset{\upsilon =1}{\sum }}\frac{\left|D^{\upsilon }\right|}{D}. \end{array}$$

Therefore, according to the Gini index, we can judge which attribute is the best split attribute. It is determined by deducting from one the total of the squared probability for each class. In contrast to information gain, which promotes smaller partitions with unique values, it favors bigger partitions and is simpler to implement. For a split, a feature with a lower Gini index is picked. The Gini coefficient's fundamental flaw as a gauge of income inequality is that it is unable to distinguish between various types of imbalances.

(7) $$\begin{array}{c} \text{Gini}\left(D\right)=1-\overset{n}{\underset{i=1}{\sum }}. \end{array}$$

The characteristics of media fusion recognition algorithm are content fusion and channel fusion, media technicalization and omnipotence, intensive production of content production, and national writing. Vision fusion is the process of fusing together various input images into a single set of images. With the continuous development of multifunction and integration of media, a single media such as mobile phone can keep abreast of major events and minor events in the world at any time, and everyone can talk and communicate with people he has known all his life [27]. The media fusion recognition algorithm's parameters are all interconnected. When we train the model, the loss of backpropagation acts on both the first module and the second module. At the same time, the online behavior track module will be adjusted according to the feedback of the students' basic characteristics module, which will also be affected by the characteristics of students' online behavior track. Knowing your high school kids will also enable you to foresee or recognize any potential personal problems. If you are familiar with your students, you will be able to tell when they are acting oddly or are depressed. If you observe this, you can step in to support them or refer them to where they can receive assistance. According to research, tracking for conventional teaching has little effect on the academic performance of low- and average-ability kids, but it has a significant positive impact on gifted students who participate in tracks created especially for gifted and talented students. The feature comparison of media fusion recognition algorithm is shown in Figure 2.

The media fusion recognition algorithm is a new model under the diversified development of information transmission. It effectively combines traditional media such as newspapers and television stations with new media communication channels such as handheld intelligent terminals and computer terminals, and generates various forms of information products through centralized processing and resource sharing, and then spreads them to the audience by relying on various platforms [28]. We use the long-term and short-term memory network to capture the time-dependent relationship between the days. RNN of the Long Short-Term Memory (LSTM) type can learn order dependence in sequence prediction issues. The calculation is as follows:

(8) $$\begin{array}{c} O_{t}=\sigma \left(W^{\left(9\right)}*\left(h_{t-1},x_{t}\right)\right), \end{array}$$

(9) $$\begin{array}{c} h_{t}=o_{t}*\tanh\left(C_{t}\right). \end{array}$$

Where

*h*_*t*_ represents the hidden state of output on day *t*,

*h*_*t*−1_ represents the hidden state of output on day *t* − 1,

*x*_*t*_ represents the input on day,

*C*_*t*_ represents the cell state on day *t*, and

*σ* and tanh are activation functions.

The result obtained is the output of the online behavior track module, as shown in the formula, where

*s* ^*tra*^ represents the online track result and

*h* ^*T*^ represents the online hidden status in *T* days.

(10) $$\begin{array}{c} s^{tra}=f\left(W^{\left(10\right)}*h^{T}\right). \end{array}$$

Connect the outputs of the two modules together as the input of the next layer of fully connected neural network. The connection operation is shown in the formula, where

*s* ^*base*^ represents the basic characteristics, and

*s* ^*base*^ is the summary of the students' online trajectory mode information and basic attribute information.

(11) $$\begin{array}{c} s^{\text{concat}}=f\left(W^{\left(11\right)}\text{concat}\right). \end{array}$$

Our goal is a binary classification problem. The simplest kind of machine learning task is binary classification. Binary classification seeks to group data items into one of two categories, such as 0 or 1, true or false, will survive or will not survive, and have blue eyes or not. We use sigmoid function to convert the output result into a value between 0 and 1.

The change of language form has given birth to the change of media form. From a diachronic perspective, written language has developed into digital language. Human beings have experienced the stage of print media and electronic media. Usually we call the printed media, such as newspapers and magazines, which release news or information on paper as the carrier “print media”. The in depth and effective research on audience psychology is an important link to realize the value transformation of animation industry resources. A participant experiences an audience effect when they act differently because they think someone is watching them. One of the earliest psychological effects was the focus of extensive research in the 1960s and 1970s but has subsequently attracted less attention. Only by adapting to the environment and changing creative ideas and strategies can we better develop university students' psychological education. The media fusion recognition algorithm has brought great changes to university students' psychological education in the form of communication, production, and experience. Although the global print media has been impacted by electronic media, especially the Internet, print media is also strengthening cooperation with electronic media. The two media are showing a state of “integration and win-win”, and neither of them is indispensable.

### 3.2. University Students' Psychological Health Standards

University students' healthy psychology should meet the following standards: first, normal intelligence. Intelligence is the sum of a person's observation, memory, imagination, thinking ability, and operation ability. Normal intelligence is the most basic psychological condition for a person to study, live, and work, the psychological guarantee for people to adapt to the environment and seek survival and development, and the primary standard for university students' psychological health. In the process of carrying out psychological health education, teachers should first master various communication technologies, constantly improve their media literacy, keep in close contact with students by using various new media, understand the psychological characteristics of university students, reveal the law of their psychological changes, and truly become their guides. Our emotional, psychological, and social well-being are all parts of our mental health. It influences our thoughts, emotions, and behaviors. Additionally, it influences how we respond to stress, interact with others, and make good decisions. Every period of life, from childhood and adolescent years to maturity, is vital for mental health. Many students' reaction is that they do not have much to say with their parents, even if they write letters, they are basically due to substantive problems such as economic supply, material supplement rather than emotional communication. Although I realize that it should not be like this, it is a common state of mind that I am too lazy to write. On the contrary, the letters between lovers are getting thicker and thicker, and the phone calls are getting denser and denser, which is in sharp contrast. On the whole, students are basically satisfied with their parents, and they also affirm their affection. However, they have fewer returns and confidently believe that their parents do not seek returns. The self-management and control of university students' emotions is not only an important part of their physical and psychological health, but also a necessary condition for their self-development and personality growth, and the basis for them to face setbacks and adapt to the environment. The network infrastructure in colleges and universities is becoming more and more perfect, which provides favorable conditions for university students to use the network. Most university students cannot resist the numerous and complicated information.

They are not only concerned about the knowledge function of the network, but also have a strong interest in its entertainment function and news function. All this information will have a negative impact on the development of university students' independent thinking ability, right and wrong discrimination ability and rational thinking ability. This unique cultural and humanistic atmosphere on campus has fostered the development of students' emotions. This is not only a problem in interpersonal communication, but also the relationship with love. The humanistic perspective places a strong emphasis on each person's intrinsic worth, the significance of human values, and the creative and active character of people. The approach is upbeat and emphasizes how admirable it is for people to be able to endure suffering, agony, and hopelessness. On the edge of emotion, many students are wandering. When dealing with personal emotional problems, they cannot see friendship and love clearly, and they cannot grasp the scale of communication between male and female students well. I aim to value friendship and unintentionally let it disappear. What university students need most is good media literacy. Media literacy refers to the ability to acquire and understand media information in various environments, which is an organic part of university students' moral quality. Whether one's mood and feelings are stable and optimistic is the main sign of one's psychological health. Positive emotions such as happiness, optimism, cheerfulness, and satisfaction are always dominant in mentally healthy people. Although there are negative emotions such as sadness, sorrow, and anger sometimes, they generally do not last long; strive to meet their own needs within the scope permitted by the society; I am satisfied with everything I can get, and I am always cheerful and optimistic. What university students do not like most is blunt preaching and boring theoretical knowledge. In order to prevent them from forming contradictory psychology and rebellious psychology, psychological health teachers should take what university students are most concerned about or the people and things that happen around them as the starting point of psychological health education, and pass on psychological health knowledge to students with vivid language, vivid cases, and various forms.

Suicide frequently results from a variety of emotional issues, academic strain, or interpersonal hurdles. Everybody is at a different age and has different perspectives on the world. Pressure from various sources will result in excessive behavior, especially in 16 to 28-year-old youths, once they pass the breaking point. They lack the minimum “ability to reduce pressure” in the face of pressure, leading to the lack of motivation in the face of pressure and the tragedy that should not happen. All sectors of society must pay full attention to this problem from the perspective of recognition and action, and help “heaven's favorite” to stay away from “depression” and regain a sunny and healthy mentality. Educators should consciously and systematically cultivate students' media literacy, and enhance their ability to resist bad information. Psychologically healthy university students have strong emotional management and adjustment ability, stable mood, optimism, exuberance, and full of hope for life and future. Be able to properly express and control emotions, vent their emotions reasonably, and correctly handle emotions such as joy, anger, sadness, and joy in life. Finally, it cannot be ignored that we should mobilize the wider social forces, publicize the knowledge of psychological health by using TV, radio, newspapers, magazines and other media; widely publicize the knowledge of psychological health, set up special columns, hotlines and consultation services, and improve university students' psychological health awareness. With these powerful guarantees, our psychological health education will really be implemented. In the college stage, the individual's self-awareness is gradually enhanced, but for a long time, they have not formed a solid image about themselves, and their self-awareness is not stable enough. Seeing problems is often one-sided and subjective, coupled with psychological vulnerability. Once they encounter temporary setbacks and failures, they are often discouraged and timid. In front of teachers, they often hide their true emotions and do not want to easily reflect their true psychological state. Impulsiveness and internalization interweave, which makes college students have intense psychological conflicts at this stage. Under the premise that college students are not rich in social life experience, they are likely to have strange and extreme thoughts and behaviors, which should also be paid attention to.

## 4. Results and Analysis

### 4.1. Psychological Health Data of University Students

This study examined the internal consistency reliability of each factor, Cronbach coefficient and split half reliability. The internal consistency of a set of items, or how closely connected they are to one another as a group is measured by Cronbach's alpha. It is regarded as a gauge of the stability of the scale. The measure is not necessarily unidimensional if alpha has a “high” value. When determining split half dependability, the complete collection of items related to an interest construct is divided in half, and the findings from the two resulting subsets of items are compared as shown in Table 1.

It can be seen from Table 1 that the reliability of all factors and the total questionnaire has reached the general standard and the overall level has reached an acceptable level, indicating that the questionnaire has good reliability.

This experiment further analyzes the differences of psychological resistance scores of university students in the process of psychological education. The experiment was conducted in freshmen, sophomores, juniors, and seniors, respectively. The change trend of each grade in each dimension is shown in Figure 3.

From Figure 3, we can see the difference of psychological education impedance of university students in different grades and the changing trend of each factor dimension. From the vertical point of view, the psychological education impedance of university students is junior, freshman, sophomore, and senior from high to low in grade. Horizontally, the scores of juniors in 17 and 18 dimensions are higher than those of the other three grades, and the juniors score the highest.

This experiment is based on the category scoring standard: the first category of total scores is those who may have mental disorders or mental diseases; the second category of total score is those who may have general psychological problems; the third type is the experimental analysis of the number of normal students, and the experimental results are shown in Figure 4.

As can be seen from Figure 4, the average proportion of “post-90s” university students with normal psychology is 88.56%; the average proportion of university students with general psychological problems is 77.25%; and the average proportion of university students with mental disorders or mental diseases is 75.32%. From this experiment, it can be explained that at present, university students still account for a large proportion of mental diseases. It is necessary to pay attention to the psychological health problems of university students. We believe that cultivating university students with the basic characteristics and basic spiritual elements of a sound personality should establish the ideal goal of personality as an ideal model of a sound personality for university students.

1502 test papers were analyzed. Variance analysis was conducted on each dimension factor to test whether there were differences in gender, grade, discipline, and source, so as to specifically explore the characteristics of resistance in the process of university students' psychological education. The test results of grade difference of university students' psychological education impedance are shown in Table 2.

From Table 2, we know that *F* = 3.677 and *P* = 0.013, which indicates that there are significant differences in various factors of impedance in the process of psychological education of university students in different grades. Back testing found that freshmen scored significantly higher than sophomores and juniors. Therefore, attaching importance to the shaping of university students' sound personality is the inevitable choice made by modern education facing the future society, and it is a new “Hope Project” with strategic significance, which has great and far-reaching significance.

### 4.2. An Analysis of University Students' Psychological Health

In order to further discuss the influence of features on the experimental results, the following feature set training models are used for experiments. The experimental results are shown in Table 3.

It can be seen from Table 3 that the experimental results of feature set I are the best. Secondly, with the reduction of feature types, the experimental results gradually become worse, especially in feature set IV, because a large number of consumption features have a great impact on the experimental results. The experimental results show that various behavioral data can improve students' cognitive effect on mental health problems. Only by cultivating and bringing up a large number of high-quality talents who can survive and create, adapt to the fierce social competition, withstand the test of difficulties and setbacks, and have good mental health and personality, can provide a reliable “cornerstone” and guarantee for the development of the future society.

This experiment analyzed the differences of psychological health resistance scores of college students in the process of psychological education. Anxiety, despair, and stress are the most prevalent problems among their college student patients, according to mental health professionals at colleges and universities. Up to 41% of college or university students were thought to exhibit depressive symptoms. The experiment was conducted in grade one, grade two, grade three, and grade four. The average change of each factor score of each grade is shown in Figure 5.

It can be seen from Figure 5 that the average changes of the scores of various factors in university students' psychological education. When the number of experiments reaches 26, the average of freshmen, sophomores, juniors, and seniors is 5.98, 5.12, 5.86, and 6.58, respectively. It can be concluded that the first one is senior, followed by freshman, junior, and sophomore.

This experiment compares and analyzes university students' personality questionnaire of different genders. The experimental results are shown in Figure 6.

As can be seen from Figure 6, the total scores of “post-90s” college boys are extremely significantly different from those of “post-90s” college girls, and the scores and total average scores of girls in various projects are higher than those of boys, which show that the psychological health level of girls is lower than that of boys. Improving university students' personality education is also the need of social civilization and progress. Modern society is driven by reform, and the torrent of reform permeates all levels of social life.

Reform is inseparable from creativity and competition, which are the most prominent features of modern social development. This social feature requires that education should be transformed from “education for the formation of academic qualifications” to “education for adults focusing on the formation of personality”. The test of gender differences in psychological education of university students is shown in Table 4.

It can be seen from Table 4 that gender differences are an important aspect of psychological research. From Table 4, it can be seen that there is no significant gender difference in various factors in the process of university students' psychological education.

In this experiment, the accuracy of university students' psychological health is compared according to different algorithms. Ant colony algorithm, decision tree algorithm, and this method are used, respectively. The experimental results are shown in Figure 7.

As can be seen from Figure 7, in the process of comparing the accuracy of university students' psychological health, this method has the highest accuracy, up to 99.25%, followed by the decision tree algorithm, up to 80.53%, and finally the ant colony algorithm, up to 75.25%. Therefore, this method is more conducive to the study of university students' psychological health. The education of healthy personality of university students refers to the education aimed at developing students' psychological quality and cultivating healthy personality to meet the needs of modern society. Through personality education, students' healthy personality can be cultivated. Considering the value of personality education from a broader perspective, it also plays a great role in promoting and sublimating social civilization. It is an important aspect of reconstructing contemporary national spirit.

## 5. Conclusions

As outstanding young college students, their mental health growth and success are related to the future and destiny of the country. In the process of everyone's life, no matter how the world develops and changes, they should face it positively and optimistically and learn to communicate with others to reduce their own pressure. People are highly social, therefore, if they do not communicate, they'll develop autism and become more reclusive. In the process of comparing the accuracy of college students' mental health, the accuracy of this method is the highest, up to 99.25%, followed by the decision tree algorithm, up to 80.53%, and finally the ant colony algorithm, up to 75.25%. Therefore, this method is more conducive to the study of college students' mental health. Through the media fusion recognition algorithm, we should fully respect the current situation of students and their current values, outlooks on life, and rights; actively guide them to identify, affirm, and like themselves; establish self-confidence and achievement motivation, and establish a correct moral outlook, outlook on life, and sense of diligence. Any social moral system should establish the ideal personality as the direction and objective of people's moral development in the new era as we pursue the ideal personality under the notion of media integration. It injects rich spiritual power resources into people's all-round development and regulates the direction of people's development. In future, new technologies are developed which helps to identify accuracy of college students' mental health efficiently.

## Figures and Tables

**Figure 1:** Flow chart of identification algorithm of students' psychological health problems based on media fusion.

**Figure 2:** Comparison of features of media fusion recognition algorithms.

**Figure 3:** The changing trend of grade 3 in all dimensions.

**Figure 4:** Comparative analysis of university students' psychological problems.

**Figure 5:** Average change of scores of each factor in grade 5.

**Figure 6:** Comparison of psychological health level of university students of different genders.

**Figure 7:** Accuracy of university students' psychological health under different algorithms.

**Table 1:** Reliability coefficient of university students' psychological education impedance questionnaire.

Reliability index	Factor 1	Factor 2	Factor 3	Factor 4	Factor 5	Overall questionnaire
Reliability	0.821	0.714	0.613	0.675	0.662	0.785
Split half reliability	0.775	0.682	0.641	0.724	0.657	0.683

**Table 2:** Grade difference test of psychological education impedance of university students.

Grade	Average value	Standard deviation	*F*	*P*
Freshman	84.9454	8.05572	3.677	0.011
Sophomore	83.1750	9.56624		
Junior	83.6214	8.58726		
Senior	84.9404	8.89577		

**Table 3:** Experimental results of four different feature combinations on the media fusion recognition algorithm model.

Dataset	Precision	Recall	F1 measure
I	0.72	0.74	0.71
II	0.68	0.72	0.72
III	0.65	0.67	0.66
IV	0.61	0.56	0.58

**Table 4:** Gender difference test of university students' psychological education.

Gender	Average value	Standard deviation	*F*	*P*
Male	84.1356	8.55405	0.457	0.498
Female	83.8113	9.12143		

## Data Availability

The data used to support the findings of this study are available from the corresponding author upon request.
